The article "Perioperative Management and Long-Term Outcomes in Ocular Cicatricial Pemphigoid Patients Undergoing Cataract Surgery" was retracted in 2023. Reasons: signs of a paper mill; suspected computer-generated content; unreliable results or conclusions; concerns about the data.

# Perioperative Management and Long-Term Outcomes in Ocular Cicatricial Pemphigoid Patients Undergoing Cataract Surgery

**DOI:** 10.1155/2022/2496649

**Published:** 2022-04-30

**Authors:** Yuan He, Zhuoya Quan, Ruixue Zhang, Zhi Ji, Jun Jia, Huifeng Liu, Chuntao Zhang, Beilei He, Yuan Ren, Yun Feng

**Affiliations:** ^1^The Second Affiliated Hospital of Xi'an Medical University, Eye Center, Ocular Immunology and Inflammation Institute, Shaanxi Provincial Clinical Research Center for Ophthalmology, Xi'an 710038, China; ^2^Department of Ophthalmology, Peking University Third Hospital, Beijing Key Laboratory of Restoration of Damaged Ocular Nerve, Peking University Third Hospital, Beijing 100191, China

## Abstract

**Objective:**

To observe the outcomes of cataract surgery in ocular cicatricial pemphigoid (OCP) patients and explore routine perioperative medical treatments.

**Design:**

Retrospective case series.

**Methods:**

Fourteen eyes of 8 patients were included in the study. Foster's stage 1-4 OCP patients were given human intravenous immunoglobulin, whereas patients with active inflammation were treated with prednisone tablets and methotrexate. Those who were intolerant to methotrexate and had severe inflammatory symptoms were treated with cyclophosphamide. Cataract surgery was performed for all patients after three months of systemic treatment under stable conditions. The conjunctival biopsy was evaluated by immunofluorescence microscopy. Then, patients were divided into individuals with or without ankyloblepharon. Records were reviewed for OCP stage, type of surgery, best-corrected visual acuity (BCVA), Schirmer I test, corneal fluorescein sodium staining, meibomian gland coloboma range, and ocular surface disease index (OSDI) scores. Follow-up was for the duration of taking topical and systemic medication.

**Results:**

Nine female (64.29%) and 4 male (35.71%) eyes were diagnosed with OCP by biopsy. The mean follow-up time was 60.64 ± 35.62 months. Thirteen eyes (92.86%) of 7 patients underwent phacoemulsification. One eye underwent phacoemulsification combined with amniotic membrane transplantation. The intracapsular extraction of cataract was applied to one eye. The BCVA improved significantly in all the patients, which remained stable until the last follow-up. The Schirmer I test was higher than that before the surgery. Corneal fluorescein sodium staining after surgery showed a decrease in score compared to the preoperative score. The BCVA of the patients after surgery increased significantly. The OSDI scores of patients with ankyloblepharon were significantly higher than for those without it. Postoperative symblepharon showed no significant difference compared to the preoperative symblepharon.

**Conclusions:**

In this series, OCP patients with cataracts were able to undergo phacoemulsification surgery, whereas routine use of immunosuppression and closed postoperative follow-up were necessary.

## 1. Introduction

Mucous membrane pemphigoid (MMP) is a systemic autoimmune bullous skin disease which mainly affects mucosal tissues, such as the conjunctiva, nasal cavity, oropharynx, esophagus, trachea, skin, and genitals [1]. Approximately 70% of patients with ocular damage as the main clinical symptom have bilateral [2], asymmetric, and chronic progressive fibrosis and inflammatory conjunctivitis, known as ocular cicatricial pemphigoid (OCP) [3]. According to relevant reports, OCP is a rare and potentially blinding disease. One of its characteristics is that it destroys the adhesion between the conjunctival epithelium and the subepithelial tissues, thereby causing the subepithelial tissues to form blisters [2]. The incidence rate of OCP is 1-5/60,000, mainly in women (male to female ratio is approximately 1 : 2). The average age of onset of patients was 65 years old, and all ethnic groups were roughly the same [4, 5]. Patients affected by this autoimmune disease will eventually develop conjunctival scarring. If the patient does not receive proper treatment or is not treated, it may cause ocular corneal opacity and permanent vision damage and loss [6]. OCP is an autoimmune chronic cicatricial conjunctivitis, and abnormal immune system regulation is an important feature of OCP [4]. Thus, ocular MMP treatment guidelines are designed to control immune-mediated inflammatory diseases, prevent fibrosis, and manage ocular surface diseases [7]. Mycophenolate mofetil, azathioprine, and methotrexate can be used for the treatment of moderate disease. Of these drugs, mycophenolate mofetil had the best safety profile and was well tolerated, with the lowest withdrawal rate among the drugs used. The recommended dose is 1 gram twice daily, and the treatment can be controlled in 59% of patients [8, 9].

Surgical operations may stimulate the patient's immune response, which had entered the cessation period of inflammation [10]. Such patients should be treated with preservative-free artificial tear eye drops, topical steroids, or immunosuppressants. In the stable period of inflammation, OCP and Stevens-Johnson syndrome (SJS) or toxic epidermal necrolysis (TEN) are safe for cataract extraction [11, 12]. Cataracts are visual impairments caused by decreased transparency and refractive power of the lens. When cataracts become obvious, surgery is the only certain treatment. Patients without other complications usually have excellent postoperative vision after cataract surgery [13]. The reported success rates for improved visual acuity in age-related cataract surgeries range from 91% to 98.5% [14, 15]. When cataracts are associated with other ocular surface diseases, such as Steven-Johnson syndrome (SJS), OCP, silkworm corneal ulcer, spring keratoconjunctivitis, and limbal stem cell deficiency, the prognosis of visual quality is rarely reported [15]. Puranik et al.'s study reported the outcomes of cataract surgery in ocular cicatricial pemphigoid and found that cataract surgery could be safely performed with no major intra- or postoperative complications [11]. However, OCP patients often present common causes of cataracts, which may result in visual loss through aging, medication-induced or complex cataracts. Age-related cataracts are more common in OCP patients because they tend to occur at an older age [6]. Drug-induced cataracts may be caused by local and systemic steroids used to treat conjunctival inflammation, and complex cataracts may be caused by uveitis associated with keratitis [16]. Vision improvement of such patients after cataract surgery may not be comparable to that of patients with senile cataract alone. Many studies have shown that surgical interventions such as cataract removal often trigger excessive inflammation in the eyes of OCP patients, leading to disease deterioration. In most patients, it is difficult to observe cataracts through the opaque cornea, which could increase the risk and difficulty of the surgical process [17]. At the same time, the risk of complications after surgery is also increased with a higher degree of scar adhesion or aggravated corneal disease after surgery. Previous studies have shown that cataract surgery can achieve certain success after complete control of conjunctival inflammation before surgery [18]. However, due to the progressive scar formation of the disease itself, the benefits of improved vision are short-lived [17].

The significance of cataract surgery in patients with OCP, the opportunity for surgery, and the choice of methods have always been controversial. Improper perioperative medication can aggravate existing ocular symptoms in OCP [15]. Therefore, the motivation and purpose of our study are to indicate the safety and effectiveness of such patients after cataract surgery and to provide guidelines for clinical research and treatment in OCP patients through evaluating ocular manifestations and symptoms of OCP stage, BCVA, Schirmer I test, corneal fluorescein sodium staining, meibomian gland coloboma range, and OSDI scores after surgery. We suggest that the routine use of immunosuppression and postoperative close follow-up are necessary.

## 2. Methods

### 2.1. General Data

The study was a retrospective cohort case study. A total of 14 eyes from 8 patients diagnosed with OCP who underwent cataract surgery in the Department of Ophthalmology, at the Second Affiliated Hospital of Xi'an Medical University from 2010 to 2018, were included and followed up for at least 2 years. The described research adhered to the tenets of the Declaration of Helsinki, and Ethics Committee approval of the Second Affiliated Hospital of Xi'an Medical University was obtained. All patients met the diagnostic criteria of ocular cicatrix pemphigoid disease with lens opacity [19]. The basic information of the patients and the detailed medication history related to the disease were collected. Every patient underwent evaluation, including BCVA (LogMAR), slit lamp examination, Goldmann applanation tonometry, and indirect fundoscopy before surgery. Ocular surface disease index (OSDI), Foster's staging system (Table 1), stage of keratopathy (Table 2), stage of the symblepharon degree (Table 3), corneal sodium fluorescein dyeing (Table 4), score of meibomian gland coloboma range (Table 5), aqueous flare, and Schirmer I test were compared before and after surgery. The surgical procedure, serological markers, and postoperative complications were recorded for each patient.

Inclusion criteria: (1) patients who met the diagnosis of OCP based on ocular manifestations, with ocular symptoms including red eyes, blepharospasm, lacrimonia, photophobia, decreased vision, burning, foreign body sensations, itching, and heavy eyelids associated with dry eye. (2) A slit lamp was used to evaluate the ocular lesions in detail. Trichiasis, dichiasis, blepharoglandular dysfunction and blepharitis, conjunctival congestion, papillary hyperplasia, and follicular formation were observed. In severe cases, conjunctival keratosis with subepithelial fibrosis, fornix shortening, and conjunctival scarring may be present. (3) Local eye conjunctiva was taken for lab examination. Direct immunofluorescence microscopy showed linear fluorescence along the conjunctival epithelial basement membrane region. (4) In accordance with the diagnostic criteria of cataract (LOCS III), after the pupil was dilated at least 5 mm, the lens was examined by ophthalmoscope or slit lamp microscope with the opacity accompanied by painless vision loss. (5) Consent for the operation was provided and the informed consent was signed. (6) The cataract surgery indications were met. (7) All patients were diagnosed for the first time without taking relevant therapeutic drugs. (8) All patients were followed up with for more than 2 years. Exclusion criteria: (1) patients with other serious physical or tumor diseases; (2) people with mental illness; (3) patients with insufficient medical records; (4) patients with follow-up less than 2 years.

### 2.2. Treatment Protocols

Patients with Foster's stages I-IV were given 2-3 g/kg human immunoglobulin (IVIG) systemic intravenous injection within 4-5 h per day and divided into three equal parts for at least three days. Cataract surgery was performed after ocular surface inflammation was in the quiescence phase (no conjunctival congestion or secretions and no progress in subconjunctival scar formation). Patients with active inflammation are routinely treated with prednisone tablets (starting at 1 mg/kg/d) in combination with methotrexate, with the doses ranging from 5 to 10 mg/week. Folic acid (5 mg) was taken orally the next day after methotrexate administration, to reduce its adverse reactions. Cataract surgery was performed after 3 months when the inflammation was stable. Methotrexate intolerance and stage IV fosters were treated with prednisone tablets (starting dose 1 mg/kg/d) combined with cyclophosphamide (1-2 mg/kg/d).

Prednisone tablets (1 mg/kg/d) were taken orally for all patients 1 week before surgery, and levofloxacin eye drops were given to the eyes 3 days before surgery, 4 times per day. Compound tropicamide eye drops (0.5%) were applied to the eyes to fully dilate the pupils before surgery. The dosage of prednisone tablets was reduced after 4-16 weeks when the inflammation was stable, by withholding one to two tablets every two to four weeks until the dosage was 10 mg daily, and then reduced to one tablet every 4-8 weeks. Prednisone was withdrawn until the condition of OCP patients was stable. The patients who were treated with immunosuppressants before surgery continued to take them after surgery.

### 2.3. Biological Sample Processing

A 2 mm × 6 mm inferior fornix of conjunctiva sample was obtained with sterilized smooth forceps and ocular surgical scissors after topical anesthesia for cataract surgery. The conjunctival sample was divided into two equal parts: one used for immunofluorescence microscopy and the other for hematoxylin-eosin (HE) staining. The samples were inserted into optimal cutting temperature compound (OCT) for embedding and quickly in liquid nitrogen. After quick freezing, the tissues were cut into serial sections with a cryostat at minus 20°C and stored for subsequent testing.

### 2.4. HE Staining

The slices were incubated at room temperature and stained with hematoxylin for 5 min. The slices were then differentiated in 1% hydrochloric acid ethanol for a few seconds and dehydrated with 95% alcohol for 30 s. The same procedure was used for eosin alcohol staining solution for approximately 3 min. The excess dye was rinsed with water and differentiated with 85% alcohol. The slices were successively dehydrated with different concentrations of alcohol. Finally, the slices were added to xylene to make them transparent and sealed with neutral gum and then were examined with a light microscope (Olympus, Japan) and photographed with a digital camera.

### 2.5. Immunofluorescence Microscopy

After cryoembedding at -20°C, the slices were ventilated to remove water vapor, fixed with 4% paraformaldehyde fixing solution, and washed with PBS three times. After the antigens were heated, they were naturally cooled at room temperature and incubated with goat serum for 1 h. Anti-IgA (1 : 100, Abcam, UK), IgG (1 : 300, Abcam, UK), and IgM (1 : 1000, Abcam, UK) antibodies were then added overnight at 4°C. Fluorescence isothiocyanate- (FITC-) labeled sheep anti-human antibodies IgA, IgG, and IgM were added followed by incubation in the dark, at room temperature for 1 h. After washing with PBS, the nuclei were stained with DAPI, and the antiquenching agent was used to seal the slices. The slices were then observed under a confocal microscope (Nikon, Japan).

### 2.6. OSDI Score

According to the subjective feelings of the patients, the OSDI scoring scale [20] was used to self-test the patients. The completion of the questionnaire was carried out under the strict professional guidance of ophthalmologists in our hospital. This questionnaire contained a total of 12 questions, for example: whether the patients have photophobia, pain, and foreign body sensation and other eye discomfort symptoms; whether there was blurred vision and visual fluctuations in the daily reading, writing, driving, the use of computers and television; and whether eyes in the sand, dry, and air conditioning environment felt uncomfortable. Each question was followed by five possible answers: 0 (never experienced such symptoms), 1 (occasional occurrence of such symptoms), 2 (had such symptoms about half the time), 3 (most of the time), and 4 (this kind of symptom occurred all the time). Patients answered the questions selectively but responded to at least two items. Each score will be summarized with a score range of 0~100, calculated by the following formula: OSDI score = (total score × 25)/number of questions.

### 2.7. Follow-Up Observation Indices

LogMAR visual acuity was recorded at 1 day, 1 week, 1 month, 3 months, 6 months, 1 year, and 2 years and at the final follow-up after surgery. The conjunctiva, cornea, and anterior segment were examined with a slit lamp. Ankyloblepharon and inflammation were examined and compared with those before the operation. The OSDI score was used to distinguish between patients with normal eye and dry eye. Perioperative doses and the durations of local and systemic immunosuppressive agents were recorded. Complications before, during, and after cataract extraction and other surgical interventions were also recorded. Patients were divided into two groups according to Foster's staging system and ankyloblepharon. The first group (without ankyloblepharon) included mild to moderate patients with OCP stages I, II, and III. The second group included severe patients (ankyloblepharon group) with OCP stage IV. The changes in OSDI score, Schirmer I test, corneal sodium fluorescein staining, meibomian gland coloboma range, and BCVA were compared before and after surgery among patients with different grades at different times. Routine blood and urine examinations were performed every week. Liver and kidney function examinations were also recorded every half a month. Blood pressure and blood glucose of OCP patients were kept within normal ranges.

### 2.8. Statistical Analysis

All data were analyzed by SPSS 20.0 software. Paired sample *t*-tests were used for intragroup comparisons, ANOVA was used for intergroup comparisons, repeated measure ANOVA was used to analyze intragroup differences in OSDI scores before and after surgery, and group *t*-tests or Wilcoxon rank sum tests were used for comparisons between groups. *P* < 0.05 was considered to be statistically significant.

## 3. Results

### 3.1. Demography of Patients

Seventeen eyes of 10 OCP patients underwent cataract surgery. Two of them were inadequate after follow-up and were excluded. Finally, 14 eyes of 8 patients were analyzed, including 9 eyes of 5 female patients (64.29%) and 5 eyes of 3 male patients (35.71%). The average age of the patients was 66.11 ± 6.33 years, and the mean follow-up time was 60.64 ± 35.62 months. The shortest follow-up time was 24 months, and the longest continuous follow-up time was 120 months.

### 3.2. HE Staining and Indirect Immunofluorescence Assay

Fourteen eyes of 8 patients were diagnosed with OCP and included in this study. None of them received any treatment or took medication before diagnosis. All patients underwent conjunctival biopsy during cataract surgery. Multiple typical infiltrated immune cells, such as lymphocytes, plasma cells, and white blood cells, were observed by HE staining (Figure 1(a)). A positive result with linear direct immunofluorescence labeling (green) of autoantibodies was staining along the basement membrane zone. (Figures 1(c)–1(e)). Since the time between the binocular operations was no more than three months, conjunctival tissue was excised from only one eye of 4 patients for HE staining.

### 3.3. Other Ocular Surgeries

One eye (7.14%) was unable to undergo phacoemulsification because of severe corneal opacity, and intracapsular cataract extraction (ICCE) was finally applied (patient 5). One patient (7.14%) underwent phacoemulsification combined with amniotic membrane transplantation (patient 6). One patient with a case of binoculus (14.28%) underwent upper eyelid surgical treatment of entropion and trichiasis (patient 2).

### 3.4. Comparison of Patient Information before and after Surgery

Foster's stage, corneal fluorescein sodium staining, and meibomian gland coloboma range did not change pre- and postoperatively (Figures 2(a)–2(d)).  Table 6 shows the basic information of preoperative OCP patients. Six patients underwent binocular cataract surgery (12 eyes, 85.71%), and two patients underwent monocular cataract surgery (2 eyes, 14.29%). The BCVA of patient 5 was light perception preoperatively. The BCVA of patient 8 was 0.4 in the right eye and 0.5 in the left eye. For the Schirmer I test, 9 eyes (64.29%) were hyposecreted before the operation, and 6 eyes (42.86%) were dry eyes. Foster's staging system, stage of keratopathy, stage of the symblepharon degree, and score of meibomian gland coloboma range after operation were very stable compared with those before operation, and there was no significant difference between pre- and postoperative states Table 7.

Compared to the preoperative values, the BCVA of all patients improved to varying degrees after surgery. The Schirmer I test and corneal fluorescein sodium staining were not performed within 3 months after surgery to avoid ocular infection. The postoperative results 3 months after surgery are shown in Table 8. Compared with one week after the operation, the BCVA of 5 eyes (35.71%) was still improving. The aqueous flare disappeared in some patients, which may be related to the postoperative fade of corneal edema. The Schirmer I test showed that only 4 eyes (28.57%) remained hyposecreted after the operation, and there were no dry eyes.  Table 9 analyzes the results of BCVA and Schirmer I test after operation in six months. Between 3 months and the final follow-up time, no changes in aqueous flare, keratopathy, symblepharon degree, or meibomian gland coloboma range were observed (Table 10). The BCVA in 2 eyes of one patient (14.29%) after the operation was 0. The BCVA improved by 7 lines in one eye of one patient (7.14%). There was no significant difference in the existing Foster's stage postoperatively compared to preoperatively.

### 3.5. Patient's Antibody Detection, Types, and Complications

The patient's surgical types, serological markers, and early and late complications before and after surgery are summarized in Table 11. Pemphigoid antibodies can be detected in the serum of all patients. Patient 2 (12.5%) showed a positive result for rheumatoid factor. Ten eyes (71.43%) underwent phacoemulsification and intraocular lens implantation. Three eyes (21.43%) were without intraocular lens implantation. One eye (7.14%) did not receive regular medication one year after ICCE and developed progressive conjunctival hyperemia 24 months later. Conjunctival complications occurred in 5 eyes (35.71%) after surgery, manifested as conjunctival hyperemia, which disappeared after 3 days. Corneal edema occurred in 5 eyes (35.71%). After the application of hypertonic saline eye drops and recombinant bovine basic fibroblast growth factor eye gel, corneal edema disappeared. Two patients with 2 eyes present (14.28%) did not take medicine regularly after the operation and their cornea neovascularization was worse than preoperation, but the OCP stage did not improve.

### 3.6. The Medicine of Perioperative Period

All patients took oral immunosuppressive agents at the beginning of treatment. Seven of them received oral methotrexate (87.5%), and one patient received oral cyclophosphamide (12.5%). All patients were intravenously injected with immunoglobulin, and prednisone tablets were taken one week before the operation. The patients stopped taking oral prednisone three months postoperation. Immunoglobulin was discontinued after the operation. Patient 1 was given cyclosporine eye drops before the surgery, and recombinant human interferon *α*-2 injection (I*α*-2aI) was used for 2 weeks after surgery. Fluorometholone eye drops were applied until the ocular symptom condition was stable (Table 12).

### 3.7. Comparison of Eye Conditions

The BCVA (Table 13, Figure 3) was lower than 2 in only 3 eyes (21.43%) before the operation, while the number of patients was increased to 11 eyes after the operation (78.67%). The BCVA was significantly improved after the operation in all patients compared to preoperative values (Table 14, Figure 4(a)) (*P* < 0.001). The difference between the BCVA between the with and without ankyloblepharon groups was statistically significant on the first day after surgery (*P* < 0.05). There was no statistically significant difference in the subsequent days (Table 15, Figure 4(b)). Schirmer I test numerical value in all postoperative patient increased and improved compared to preoperative (Table 14, Figure 4(c)) and was statistically significant (*P* < 0.01). There was no statistical significance in the comparison of the difference of Schirmer I test between the group with or without ankyloblepharon after operation (Table 16, Figure 4(d)). The positive rate of corneal sodium fluorescein dyeing at 6 months, 1 year, 2 years, and the final follow-up time decreased significantly compared to preoperatively (Table 14, Figure 4(e)) (*P* < 0.01). The difference in corneal sodium fluorescein dyeing between the group with or without ankyloblepharon was not statistically significant after surgery (Table 17, Figure 4(f)). The meibomian gland coloboma range in all patients remained unchanged after surgery (Table 14).  Figure 5 shows the difference in OSDI score between preoperative and postoperative samples. Figures 6–8 show the preoperative and postoperative images of the partial anterior segment.

### 3.8. OSDI Questionnaire Survey Analysis

The OSDI scores of patients with OCP stages I, II, and III were significantly higher at 1 day and 1 week postoperation than preoperation. The OSDI scores of patients with OCP stage IV were higher at 1 day, 1 week, and 1 month after surgery. The score significantly increased before operation and then began to decrease until it eventually reached the same level as preoperation, but there was no statistically significant difference between each group before and after treatment (*P* > 0.05). The average OSDI scores of patients with preoperative and postoperative OCP stages I, II, and III were significantly higher than those of grade IV patients (*P* < 0.01) (Table 18).

## 4. Discussion

MMP is a skin disease with chronic, recurrent, and multisystemic autoimmune dysfunction. Inflammation and scar formation on mucosal surfaces are characteristic pathological clinical manifestations of OCP [21]. It has been reported that the visual acuity of patients with OCP combined with cataracts improves poorly after phacoemulsification [6]. The main reason for the poor prognosis of vision is the progression of the disease and subsequent scarring. Maza et al. [18] reported that twenty OCP patients received systemic immunosuppression before cataract surgery and none of the patients showed disease progression during an average of 22 months of follow-up, indicating that cataract surgery can be performed safely with complete remission of the diseases.

The commonly used immunosuppressants for OCP patients are cyclophosphamide, azathioprine, methotrexate, and dapsone. Patients should be given less effective medicines after diagnosis and gradually change a medical prescription. It has been reported that preoperative and postoperative use of artificial tears and autologous serum eye drops can help stabilize the ocular surface condition [21]. All of our patients were treated preoperatively and postoperatively. Bissen-Miyajima and his team reported that the combination of limbal and amniotic membrane transplantation for ocular surface reconstruction and cataract surgery showed a faster visual rehabilitation effect in SJS patients [22]. One eye of our patients was treated with amniotic membrane transplantation combined with cataract surgery, and the BCVA improved significantly.

According to the visual acuity statistics in our study, the postoperative BCVA was 57.14% higher than the preoperative BCVA. The BCVA of 5 of 14 eyes (36%) met the legal criteria for “blindness” before surgery, but navigated visual acuity was achieved in all eyes after surgery. This result shows that OCP patients with well-controlled inflammation can obtain good visual benefits after cataract surgery. Control of long-term medication can maintain good visual acuity. The BCVA of one patient in their right eye improved from 1 to 0.5 after 120 months of follow-up after surgery. The BCVA of the left eye improved from 1.3 to 0.6. All patients' BCVA improved postoperatively, and the *P* values were less than 0.001. The BCVA on the first postoperative day between patients with or without eyelid adhesions was significantly different. This was mainly because the patients without eyelid adhesions and cataracts had milder lesions. Phacoemulsification energy had little effect on the cornea, due to a lower probability of corneal edema after surgery and a faster recovery speed.

It has been reported that patients with dry eye have poor BCVA due to late corneal complications, endophthalmitis, and other causes after cataract surgery [23]. The Schirmer I test of our patients increased from 7.57 ± 5.39 mm to 12.64 ± 4.68 mm after surgery. The OCP stage had no effect on the Schirmer I test results. Although there was a short-term decline in postoperative results, the long-term results were gratifying. This may be because the patients paid more attention to their eyes after surgery than before. However, Schirmer I test results alone cannot evaluate dry eye symptoms of OCP patients.

The Foster stage, meibomian gland coloboma range, corneal fluorescein sodium staining, keratopathy stage, and symblepharon degree of patients did not change after surgery. Short-term complications occurred in 6 eyes of 5 patients (42.86%). After treatment, conjunctival hyperemia and corneal edema disappeared. Corneal neovascularization appeared in 2 eyes of 2 patients (14.29%) and was aggravated compared to preoperation. After immunosuppressive treatment, the symptoms were relieved without affecting visual acuity. Cataract surgery did not cause corneal surface injury and even improved after standard treatment, independent of the degree of symblepharon, also confirmed by the OSDI score scale. However, the OSDI scores of patients with ankyloblepharon were higher than those of patients without ankyloblepharon. Cataract surgery did not affect the subjective perception between the two groups of patients. The reason why the OSDI scores before and after did not improve may be because most of the patients were middle-aged and had a low demand for driving and reading. The OSDI score scale does not fully reflect the benefits of vision correction.

With the improvement of modern cataract surgery refinement and technology, cataract extraction surgery has become safer than before. The decision of whether stage IV OCP patients should undergo cataract surgery still needs to be cautiously determined. Finally, OCP patients must consider the level of vision loss caused by cataracts. Surgeons must try to balance the risk of intraoperative or postoperative complications. All patients must be followed up in time to prevent irreversible disease progression. Therefore, preoperative treatment and advanced surgical techniques by ophthalmologists are necessary.

This study still obtains some limitations; due to the fact that this is a retrospective case study, it is not allowed to randomize the patients into groups which might jeopardize the similarity of patients in groups. Meanwhile, the treatment effect of patients administered novel medicines such as rituximab during the operation period has not been evaluated which may be one of the potential therapeutic medicines that can replace immunosuppressants or other large clinical side effects for OCP patients in the future. Besides, this study had few objective evaluations of postoperative results.

## 5. Conclusion

With complete control of ocular surface inflammation, patients with a low stage of OCP could obtain greater postoperative BCVA improvement. Standardized perioperative medication and detailed surgical plans resulted in fewer postoperative adverse reactions and complications and improved patient satisfaction. After successful elimination of active conjunctival inflammation in OCP patients with systemic steroids and immunosuppressants, there was a low risk of disease activity due to surgical trauma. Since there was no conclusive evidence about the quiescent period of OCP inflammation, the best time for surgical treatment was waiting for at least 3 months after active inflammation subsided. The prospect of this study is to provide reliable efficacy and safety support for the surgical treatment of OCP patients complicated with cataract.

## Figures and Tables

**Figure 1:** HE staining and immunofluorescence assay. (a) The histology of OCP conjunctiva. Multiple infiltrating immune cells were observed in the HE-stained slides from 10 eyes of 8 patients. (b) Control group. There was no staining along the conjunctival basement membrane zone. (c–e) Positive results of brilliant IgM, IgA, and IgG fluorescent staining along the basement membrane zone.

**Figure 2:** Preoperative and postoperative stage and score of OCP patients. (a) Foster's stage I-IV. (b) Keratopathy stage 1-4. (c) Symblepharon stage 1-3. (d) Meibomian gland coloboma range score 0-3.

**Figure 3:** Preoperative and postoperative radar images of the BCVA in OCP patients. The postoperative BCVA of the standard logarithmic visual acuity chart above 0.1 was significantly increased.

**Figure 4:** The BCVA, Schirmer I test, and corneal fluorescein sodium staining preoperative and postoperative. (a) The BCVA preoperative and postoperative (compared to preoperative, ^∗^*P* < 0.001, *n* = 14). (b) The difference in BCVA between preoperative and postoperative patients (compared to the group without ankyloblepharon, ^∗^*P* < 0.05). (c) The Schirmer I test preoperative and postoperative (compared to preoperative, ^∗^*P* < 0.001, *n* = 14). (d) The difference in the Schirmer I test between preoperative and postoperative values. (e) Preoperative and postoperative corneal fluorescein sodium staining (compared to preoperative, ^∗^*P* < 0.001, *n* = 14). (f) The difference in corneal fluorescein sodium dyeing between preoperative and postoperative samples.

**Figure 5:** The difference in OSDI score between preoperative and postoperative samples. There was statistically significant difference between the group without ankyloblepharon and the group with ankyloblepharon (^∗^compared to preoperative *P* < 0.01, the group with ankyloblepharon *n* = 6, the group without ankyloblepharon *n* = 8).

**Figure 6:** Anterior segment image of the patient in the OCP stage of Foster's stage II and III. (a) Cortical and nuclear opacifications were found in the lens after dilatation before the operation of the eighth patient in the OCP stage of Foster's stage II. Sodium fluorescein staining before surgery of the eighth patient in the OCP stage of Foster's stage II, anterior segment image 1 month and 6 months after surgery. (b) Anterior segment image of the fourth patient in the OCP stage of Foster's stage III before surgery, the double frontal fornix becomes shallower preoperatively, and there are obvious symblepharons, which are especially evident in the inner and outer canthus. (c) Anterior segment image of the fourth patient in the OCP stage of Foster's stage III in 6 months after surgery. (d) Anterior segment image of the fourth patient in the OCP stage of Foster's stage III in 2 years after surgery.

**Figure 7:** The anterior segment image of the second patient in the OCP stage of Foster's stage IV.

**Figure 8:** Anterior segment image of the fifth patient in the OCP stage of Foster's stage IV. (a) Both eyes showed corneal neovascularization before surgery. (b) Anterior segment image and sodium fluorescein staining image of both eyes 2 years after ICCE surgery.

**Table 1:** The stage of ocular cicatricial pemphigoid (Foster's staging system).

Stage	Clinical feature
I	Conjunctival congestion, subconjunctival fibrosis, chronic nonspecific conjunctivitis
II	Except for conjunctival scar, the lower fornix is shortened and the corneal epithelium is punctate stained
III	Significant eyelid adhesion, especially at the epicanthus, conjunctival scar thickening, corneal infiltration, scar, neovascularization, and dry eye
IV	Eyelid adhesions, corneal epithelial keratosis, corneal neovascularization, trichiasis, eyelash disorder, rabbit eye, varus

**Table 2:** The stage of keratopathy.

Stage	Clinical feature
0	Normal cornea
1	Mild to moderate superficial punctate keratitis
2	Severe superficial punctate keratitis
3	Mild to moderate scarring and/or neovascularization
4	Severe scarring and/or neovascularization

**Table 3:** The stage of the symblepharon degree.

Stage	Clinical feature
0	No symblepharon
1	Symblepharon only involves the conjunctival surface
2	The formation of symblepharon involves less than half of the corneal surface
3	The formation of symblepharon involves more than half of the corneal surface

**Table 4:** Corneal fluorescein sodium dyeing score.

Score	Degree of dyeing
0	Nonfluorescent dyeing
1	Fluorescein dyeing sites < 5
2	Corneal fluorescein dyeing sites < 30 and ≥5 and/or dyeing range no more than 2 quadrants
3	Corneal fluorescein dyeing sites ≥ 30 and/or corneal injury area 2 quadrants or above and fusion of dyeing sites

**Table 5:** The score of meibomian gland coloboma range.

Score	Meibomian gland coloboma range
0	No coloboma
1	<1/3 proportion
2	1/3~2/3 proportion
3	>2/3 proportion

**Table 6:** Preoperative information of patients.

Patient	Age/sex	Eye	OCP	Aqueous flare	Symblepharon	Keratopathy	BCVA	Meibomian gland coloboma range	Schirmer I test
1	51/M	OD	I	0	1	3	1	1	3
	51	OS	I	0	1	4	1.3	1	4
2	68/F	OD	IV	0	2	3	2	2	18
	67	OS	IV	0	2	1	1.9	2	7
3	64/F	OD	IV	0	2	2	1.1	2	4
	64	OS	IV	0	2	4	1.4	2	3
4	72/F	OD	III	0	2	3	1.2	2	15
	72	OS	III	0	1	2	1.3	2	10
5	71/F	OS	IV	2	2	4	0.0025	3	2
6	71/M	OD	IV	2	3	4	0.005	3	3
7	65/M	OD	IV	2	2	4	0.005	3	5
	66	OS	IV	2	2	4	0.005	3	5
8	66/F	OD	II	0	1	1	0.4	1	12
	66	OS	II	0	1	1	0.5	1	15

The aqueous flare: 0: no; 1: have; 2: not clear.

**Table 7:** The postoperation outcomes of patients after one week.

Patient	Eye	OCP	Aqueous flare		Symblepharon		Keratopathy		Meibomian gland coloboma range		BCVA	
			Postoperation	Difference	Postoperation	Difference	Postoperation	Difference	Postoperation	Difference	Preoperation	Postoperation
1	OD	I	0	0	1	0	3	0	1	0	1.0	0.7
	OS	I	0	0	1	0	4	0	1	0	1.3	1.8
2	OD	IV	0	0	2	0	3	0	2	0	2.0	1.2
	OS	IV	0	0	2	0	1	0	2	0	1.9	0.4
3	OD	IV	1	1	2	0	2	0	2	0	1.1	0.8
	OS	IV	0	0	2	0	4	0	2	0	1.4	0.9
4	OD	III	1	1	2	0	3	0	2	0	1.2	0.5
	OS	III	1	1	1	0	2	0	2	0	1.3	0.3
5	OS	IV	2	0	2	0	4	0	3	0	0.0025	0.005
6	OD	IV	2	0	3	0	4	0	3	0	0.005	0.005
7	OD	IV	2	0	2	0	4	0	3	0	0.005	0.014
	OS	IV	2	0	2	0	4	0	3	0	0.005	0.014
8	OD	II	0	0	1	0	1	0	1	0	0.4	0
	OS	II	0	0	1	0	1	0	1	0	0.5	0

The aqueous flare: 0: no; 1: have; 2: not clear.

**(a):** 

Patient	Eye	OCP	Aqueous flare		Symblepharon		Keratopathy		Meibomian gland coloboma range		BCVA		Schirmer I test
			Postoperation	Difference	Postoperation	Difference	Postoperation	Difference	Postoperation	Difference	Preoperation	Postoperation	
1	OD	I	0	0	1	0	3	0	1	0	1.0	0.6	11
	OS	I	0	0	1	0	4	0	1	0	1.3	0.7	15
2	OD	IV	0	0	2	0	3	0	2	0	2.0	1.0	17
	OS	IV	0	0	2	0	1	0	2	0	1.9	0.4	11
3	OD	IV	0	0	2	0	2	0	2	0	1.1	0.8	10
	OS	IV	0	0	2	0	4	0	2	0	1.4	0.9	13
4	OD	III	0	0	2	0	3	0	2	0	1.2	0.4	18
	OS	III	0	0	1	0	2	0	2	0	1.3	0.3	16
5	OS	IV	2	0	2	0	4	0	3	0	0.0025	0.005	5
6	OD	IV	2	0	3	0	4	0	3	0	0.005	0.014	8
7	OD	IV	2	0	2	0	4	0	3	0	0.005	0.014	6
	OS	IV	2	0	2	0	4	0	3	0	0.005	0.014	5
8	OD	II	0	0	1	0	1	0	1	0	0.4	0	14
	OS	II	0	0	1	0	1	0	1	0	0.5	0	15

The aqueous flare: 0: no; 1: have; 2: not clear.

**Table 9:** The outcome of patients after operation in six months.

Patient	Eye	OCP	Aqueous flare		Symblepharon		Keratopathy		Meibomian gland coloboma range		BCVA		Schirmer I test
			Postoperation	Difference	Postoperation	Difference	Postoperation	Difference	Postoperation	Difference	Preoperation	Postoperation	
1	OD	I	0	0	1	0	3	0	1	0	1.0	0.6	11
	OS	I	0	0	1	0	4	0	1	0	1.3	0.7	15
2	OD	IV	0	0	2	0	3	0	2	0	2.0	1.0	17
	OS	IV	0	0	2	0	1	0	2	0	1.9	0.4	11
3	OD	IV	0	0	2	0	2	0	2	0	1.1	0.8	10
	OS	IV	0	0	2	0	4	0	2	0	1.4	0.9	13
4	OD	III	0	0	2	0	3	0	2	0	1.2	0.4	18
	OS	III	0	0	1	0	2	0	2	0	1.3	0.3	16
5	OS	IV	2	0	2	0	4	0	3	0	0.0025	0.005	5
6	OD	IV	2	0	3	0	4	0	3	0	0.005	0.014	8
7	OD	IV	2	0	2	0	4	0	3	0	0.005	0.014	6
	OS	IV	2	0	2	0	4	0	3	0	0.005	0.014	5
8	OD	II	0	0	1	0	1	0	1	0	0.4	0	14
	OS	II	0	0	1	0	1	0	1	0	0.5	0	15

The aqueous flare: 0: no; 1: have; 2: not clear.

**Table 10:** The outcomes of patients after operation in final time.

Patient	Eye	Time	OCP	Aqueous flare		Symblepharon		Keratopathy		Meibomian gland coloboma range		BCVA		Schirmer I test
				Postoperation	Difference	Postoperation	Difference	Postoperation	Difference	Postoperation	Difference	Preoperation	Postoperation	
1	OD	120	I	0	0	1	0	3	0	1	0	1.0	0.5	9
	OS	120	I	0	0	1	0	4	0	1	0	1.3	0.6	19
2	OD	55	IV	0	0	2	0	3	0	2	0	2.0	1.0	16
	OS	55	IV	0	0	2	0	1	0	2	0	1.9	0.4	13
3	OD	79	IV	0	0	2	0	2	0	2	0	1.1	0.8	13
	OS	79	IV	0	0	2	0	4	0	2	0	1.4	0.9	15
4	OD	82	III	0	0	2	0	3	0	2	0	1.2	0.3	19
	OS	73	III	0	0	1	0	2	0	2	0	1.3	0.3	14
5	OS	24	IV	2	0	2	0	4	0	3	0	0.002	0.05	6
6	OD	76	IV	2	0	3	0	4	0	3	0	0.005	0.014	7
7	OD	24	IV	2	0	2	0	4	0	3	0	0.005	0.014	9
	OS	31	IV	2	0	2	0	4	0	3	0	0.005	1	5
8	OD	24	II	0	0	1	0	1	0	1	0	0.4	0	15
	OS	24	II	0	0	1	0	1	0	1	0	0.5	0	17

The aqueous flare: 0: no; 1: have; 2: not clear.

**Table 11:** Antibody detection, types, and complications.

Patient	Eye	Type	Serological markers	Postoperation conjunctival complications	Postoperation corneal complications
1	OD	Phaco+PCIOL	Antibody to pemphigoid (+)	—	—
	OS	Phaco+PCIOL		—	—
2	OD	Phaco+PCIOL	Antibody to pemphigoid (+)	Conjunctival congestion	Conjunctival congestion
	OS	Phaco+PCIOL	Rheumatoid factors (+)	—	—
3	OD	Phaco+PCIOL	Antibody to pemphigoid (+)	Conjunctival congestion	Corneal edema
	OS	Phaco+PCIOL		—	—
4	OD	Phaco+PCIOL	Antibody to pemphigoid (+)	—	—
	OS	Phaco+PCIOL		—	—
5	OS	ICCE	Antibody to pemphigoid (+)	Conjunctival congestion	Neovascularization
6	OD	Phaco	Antibody to pemphigoid (+)	Conjunctival congestion	Corneal edema
7	OD	Phaco	Antibody to pemphigoid (+)	Conjunctival congestion	Corneal edema
					Neovascularization
	OS	Phaco		—	Corneal edema
8	OD	Phaco+PCIOL	Antibody to pemphigoid (+)	—	—
	OS	Phaco+PCIOL		—	—

Phaco: phacoemulsification; PCIOL: posterior chamber intraocular lens; ICCE: intracapsular cataract extraction.

**Table 12:** Steroid hormones and immunosuppressant.

Patient	Eye	Medicine				
		Preoperation		Postoperation		
		Admission	Before one week	After one week	After three months	Final
1	OD	Mtx	Mtx, IVIG, Pred	Mtx, Pred, FML, I*α*-2aI	Mtx, FML	Mtx
	OS	Mtx	Mtx, IVIG, Pred	Pred, FML, I*α*-2aI	Mtx, FML	Mtx
2	OD	Mtx	Mtx, IVIG, Pred	Mtx, Pred	Mtx	Mtx
	OS	Mtx	Mtx, IVIG, Pred	Mtx, Pred	Mtx	Mtx
3	OD	Mtx	Mtx, IVIG, I*α*-2aI, CED, Pred	Mtx, CED, Pred	Mtx	Mtx
	OS	Mtx	Mtx, I*α*-2aI, IVIG, CED, Pred	Mtx, CED, Pred	Mtx	Mtx
4	OD	Mtx	Mtx, IVIG, I*α*-2aI, Pred	Mtx, I*α*-2aI, Pred	Mtx	Mtx
	OS	Mtx	Mtx, IVIG, Pred	Mtx, Pred	Mtx	Mtx
5	OS	Mtx	Mtx, IVIG, Pred	Mtx, Pred	Mtx	Mtx
6	OD	I*α*-2bED, Pred, CED, Cyc	IVIG, I*α*-2bED, Pred, CED, FML, Cyc	I*α*-2bED, Pred, CED, Cyc	Mtx, CED, Cyc	Cyc
7	OD	Mtx	Mtx, IVIG, Pred	Pred, Mtx	Mtx	Mtx
	OS	Mtx	Mtx, IVIG, Pred	Pred, Mtx	Mtx	Mtx
8	OD	Mtx	Mtx, IVIG, Pred	Mtx, Pred	Mtx	Mtx
	OS	Mtx	Mtx, IVIG, Pred	Mtx, Pred	Mtx	Mtx

Cyc: cyclophosphamide; Mtx: methotrexate; Pred: prednisone tablets; IVIG: intravenous immunoglobulin; FML: fluorometholone; I*α*-2aI: recombinant human interferon *α*-2a injection; I*α*-2bED: recombinant human interferon *α*2b eye drop; CED: cyclosporine eye drops.

**Table 13:** BCVA distribution statistics in pre- and postoperation.

	Preoperation (*n*%)				Postoperation (*n*%)			
	>2	1.4-2	1-1.3	<2	>1	0.7-1	0.4-0.6	<0.4
BCVA	4 (28.57)	4 (28.57)	3 (21.43)	3 (21.43)	3 (21.43)	4 (28.57)	3 (21.43)	4 (28.57)

**Table 14:** Comparison of inspection result in pre- and postoperation.

Type	Eye	Statistical	Time								
			Preoperation	Postoperative day	1 week after operation	1 month after operation	3 months after operation	6 months after operation	1 year after operation	2 years after operation	Final
BCVA	14	Mean ± SD	1.5 ± 0.70	1.14 ± 0.80	0.99 ± 0.79	0.95 ± 0.74	0.93 ± 0.74	0.93 ± 0.75	0.84 ± 0.71	0.84 ± 0.71	0.84 ± 0.71
		*P*	—	<0.001	<0.001	<0.001	<0.001	<0.001	<0.001	<0.001	<0.001
		*t*	—	5.579	7.041	8.261	8.42	8.42	7.632	7.632	7.632
Schirmer I test	14	Mean ± SD	7.57 ± 5.39	—	—	—	11.71 ± 4.43	11.36 ± 4.16	11.71 ± 4.21	11.21 ± 3.79	12.64 ± 4.68
		*P*	—	—	—	—	0.001	0.006	0.003	0.019	0.001
		*t*	—	—	—	—	4.146	3.267	3.64	2.684	4.252
Corneal fluorescein sodium dyeing	14	Mean ± SD	2.86 ± 2.63	—	—	—	2.64 ± 2.50	2.29 ± 2.33	2.29 ± 2.33	2.14 ± 2.25	2.14 ± 2.45
		*P*	—	—	—	—	0.082	0.006	0.006	0.006	0.006
		t	—	—	—	—	1.883	3.309	3.309	3.238	3.238

**Table 15:** Comparison of BCVA pre- and postoperation.

	3 months after operation	6 months after operation	1 year	2 years	Final
			After operation	After operation	
Ankyloblepharon (*n* = 6)	5.00 ± 4.10	3.83 ± 4.91	4.33 ± 4.71	2.66 ± 5.47	5.67 ± 4.76
Without ankyloblepharon (*n* = 8)	3.50 ± 3.60	3.75 ± 4.20	4.00 ± 4.21	4.38 ± 5.01	4.63 ± 4.50
*F*	0.532	0.001	0.019	0.369	0.175
*P*	0.480	0.973	0.891	0.555	0.683

**Table 16:** Comparison of Schirmer I test differences pre- and postoperation.

	Postoperative day	1 week after operation	1 month after operation	3 months after operation	6 months after operation	1 year	2 years	Final
						After operation	After operation	
Ankyloblepharon (*n* = 6)	0.52 ± 0.23	0.62 ± 0.29	0.62 ± 0.29	0.67 ± 0.29	0.67 ± 0.29	0.72 ± 0.29	0.72 ± 0.29	0.72 ± 0.29
Without ankyloblepharon (*n* = 8)	0.24 ± 0.18	0.42 ± 0.24	0.50 ± 0.22	0.50 ± 0.22	0.50 ± 0.22	0.61 ± 0.36	0.61 ± 0.36	0.61 ± 0.36
*F*	6.062	1.847	0.647	1.392	0.340	0.340	0.340	0.340
*P*	0.030	0.199	0.437	0.261	0.570	0.570	0.570	0.570

**Table 17:** Comparison of corneal fluorescein sodium dyeing differences pre- and postoperation.

	3 months after operation	6 months after operation	1 year	2 years	Final
			After operation	After operation	
Ankyloblepharon (*n* = 6)	0 ± 0	−0.50 ± 0.55	−0.50 ± 0.55	−0.83 ± 0.98	−0.83 ± 0.98
Without ankyloblepharon (*n* = 8)	−0.38 ± 0.52	−0.63 ± 0.74	−0.63 ± 0.74	−0.63 ± 0.74	−0.63 ± 0.74
*F*	3.086	0.120	0.120	0.205	0.205
*P*	0.104	0.735	0.735	0.659	0.659

**Table 18:** Comparison of OSDI scores in OCP patients before and after surgery.

	Preoperation	After 1 day	After 1 week	After 1 month	After 3 months	After 6 months	After 12 months	After 24 months	Final	*F*	*P*
Without ankyloblepharon	42.86 ± 12.19	49.20 ± 7.23	49.80 ± 7.23	42.86 ± 12.19	42.86 ± 12.19	42.86 ± 12.19	42.86 ± 12.19	42.86 ± 12.19	42.86 ± 12.19	4	0.184
Ankyloblepharon	80.54 ± 9.66	86.82 ± 10.75	86.82 ± 10.75	82.64 ± 11.7	80.5 ± 9.66	80.54 ± 9.66	80.54 ± 9.66	80.54 ± 9.66	80.54 ± 9.66	4.51	0.065
*t*	4.879	5.217	5.217	5.217	4.667	4.879	4.879	4.879	4.879		
*P*	0.003	0.002	0.002	0.003	0.003	0.003	0.003	0.003	0.003		

Ankyloblepharon *n* = 6; without ankyloblepharon *n* = 8.

## Data Availability

The labeled dataset used to support the findings of this study are available from the corresponding author upon request.
